The article "Digital Industry Financial Risk Early Warning System Based on Improved K-Means Clustering Algorithm" was retracted in 2023. Reasons: signs of a paper mill; suspected computer-generated content; unreliable results or conclusions; concerns about the data.

# Digital Industry Financial Risk Early Warning System Based on Improved K-Means Clustering Algorithm

**DOI:** 10.1155/2022/6797185

**Published:** 2022-05-28

**Authors:** Xiao-li Duan, Xue-xia Du, Li-mei Guo

**Affiliations:** ^1^School of Economics &Management, Zhengzhou Normal University, Zhengzhou 450044, China; ^2^National Central City Academy, Zhengzhou Normal University, Zhengzhou 450044, China; ^3^School of Economics, Sichuan University, Chengdu, 610065, China

## Abstract

Corporate financial risks not only endanger the financial stability of digital industry but also cause huge losses to the macro-economy and social wealth. In order to detect and warn digital industry financial risks in time, this paper proposes an early warning system of digital industry financial risks based on improved K-means clustering algorithm. Aiming to speed up the K-means calculation and find the optimal clustering subspace, a specific transformation matrix is used to project the data. The feature space is divided into clustering space and noise space. The former contains all spatial structure information; the latter does not contain any information. Each iteration of K-means is carried out in the clustering space, and the effect of dimensionality screening is achieved in the iteration process. At the same time, the retained dimensions are fed back to the next iteration. The dimensional information of the cluster space is discovered automatically, so no additional parameters are introduced. Experimental results show that the accuracy of the proposed algorithm is higher than other algorithms in financial risk detection.

## 1. Introduction

Systemic financial risk refers to the risk that may endanger the stability of the entire financial system. There are many forms of systemic financial risk, the most typical of which is the financial crisis [1]. Since the 17th century, financial crises have been breaking out all over the world, and their frequency and destructiveness have increased. At present, the global financial market is still in a period of recovery and adjustment, but the international financial situation is still very grim. More importantly, with the trend and background of economic globalization, the occurrence probability and harm degree of exogenous financial risks are increasing rapidly [2].

In recent years, China's scientific and technological progress has spawned the continuous innovation and development of new financial forms. Take digital finance as an example, third-party payment services have begun to replace traditional financial sector services [3]. It has also made remarkable progress in online lending, intelligent investment, and digital insurance. But at the same time, various risk factors including loan default, fund misappropriation, false target, and even fraud also occur. Endogenous risks in China's financial system have increased significantly. Based on the characteristics of Internet technology, risks are easily contagious among different departments and regions, and may evolve into financial risks.

However, in practice, it is extremely difficult to forewarn financial risks. One of the important reasons why the traditional financial risk early warning technology does not make effective early warning is the lack of effective and timely key factors. Both academia and industry have the view that features determine the model to go online. The traditional financial risk early warning technology relies on the information and factors based on the traditional statistical data in the factor level, which itself has the lag [4]. It is averse to financial risk warning objectively. In the era of big data, the emergence of massive unstructured information provides an opportunity for financial risk warning to expand the basic information. The development of artificial intelligence in the fields of vision, natural language understanding, and other cognitive perception provides essential technical support for mining this information and ultimately forming effective and timely financial risk warning key factors [5].

Artificial intelligence is widely used in image and text data mining applications, and financial risk prediction can use this kind of technology for reference, so this paper also introduces relevant algorithms. In order to mine image information, satellite image recognition technology, optical character recognition (OCR), and natural language processing (NLP) can be used to extract information [6]. For example, targets such as crops, shipping goods, and land and sea transportation can be identified from ultra-high resolution satellite images, to give early warning of trend changes in important links of economic production [7]. OCR technology can be used to extract important information for risk audit from non-standard information, such as financial notes and transaction notes [8]. Remote sensing data of night light can be used to dynamically predict population density and urban expansion rate [9]. In addition, voice print recognition technology can be used to enhance the security of financial application scenarios and improve the effect of interactive experience, etc. [10]. For text information content, natural language processing (NLP) combined with machine learning technology can be used to complete information extraction [11]. For example, financial entities can be identified in real time from the text data of news, public opinion and forum information, the correlation of financial events can be found, and the related factors depicting economic uncertainty can be extracted [12]. From the data of annual reports, initial public offerings (IPO) prospectuses and forward-looking statements of listed companies, information such as corporate income, business development scale, and strategic tendency of corporate development can be mined [13].

However, as a new data source, image and text information have the characteristics of multisource, heterogeneous, massive, and high frequency, so it is difficult to process this kind of information [14]. (1) Multisource and heterogeneous: compared with traditional data mainly collected by governments and institutions, the release subjects and specific forms of image and text big data are diverse. There is no uniform collection standard and collection format for unstructured information, which poses a great challenge to artificial intelligence (AI) information collection and data preprocessing technology. (2) Massive data collection: limited by the cost of data collection, traditional data collection often needs the help of paper media and has a small volume. With the transfer of text information from paper media to Internet media, the cost of text data collection and transmission is greatly reduced. Terabyte data is generated every day. Screening and extracting key effective factors from massive data is not only the key point but also the difficulty of information processing. (3) High frequency: data in the traditional financial field are mostly annual, quarterly, monthly, and weekly data. However, the frequency of image and text big data can be as high as seconds or even higher, which puts forward higher requirements for the processing speed of unstructured information.

The combination of the above features makes the application of unstructured big data to financial risk warning a core challenge. How to extract valuable information accurately and effectively for risk warning from mixed multisource, heterogeneous, and high-frequency data is of great significance. In order to solve this problem, this paper proposes a financial risk prediction model based on improved K-means clustering algorithm.

The innovations and contributions of this paper are listed below.

1. The feature is divided into clustering space and noise space by transformation matrix.
2. The information density of clustering space is higher and the dimension is smaller and K-means can reduce the time consumption of each distance calculation.
3. The effect of reducing and screening characteristics can be achieved, to improve the accuracy of financial risk prediction.

This paper consists of five main parts: the first part is the introduction, the second part is financial risk prediction model based on improved K-means clustering algorithm, the third part is system design of this paper, the fourth part is the experiment and analysis, and the fifth part is the conclusion, besides there are abstracts and references.

## 2. Financial Risk Prediction Model Based on Improved K-Means Clustering Algorithm

### 2.1. Related Concepts

In order to better describe the algorithm, the following conventions are made.

For category P, the calculation formula of the *y* th dimension of its centre point is as follows.

(1) $$\begin{array}{c} P_{y}=\frac{1}{t}\sum_{x=1}^{t}I_{\text{xy}}. \end{array}$$

*T* is the amount of data of class *P*, and *I*_xy_ is the *y*-dimensional data of *I*_*x*_.

The calculation formula of Euclidean distance [2] is as follows.

(2) $$\begin{array}{c} \text{Dist}\left(I_{x},I_{y}\right)=\text{sqrt}\left(\sum_{z=1}^{w}{\left(I_{\text{xz}}-I_{\text{yz}}\right)}^{2}\right), \end{array}$$

where *I*_*x*_ and *I*_*y*_ represent the w-dimensional data object in the dataset, and *Z* represents the dimension.

The symbols used in this paper are shown in Table 1.

For cluster *X*, the dispersion matrix *S*_*x*_ is calculated.

(3) $$\begin{array}{c} S_{x}=\sum_{I\in C_{x}}\left(I-P_{x}\right){\left(I-P_{x}\right)}^{T}. \end{array}$$

For the total data, the dispersion matrix *S*_*s*_ is calculated

(4) $$\begin{array}{c} S_{S}=\sum_{I\in S}\left(I-P_{S}\right){\left(I-P_{S}\right)}^{T}. \end{array}$$

### 2.2. K-Means Loss Function

In the traditional K-means algorithm, the loss function is the sum of squares of errors, and the calculation method is as follows:

(5) $$\begin{array}{c} Y_{c}=\sum_{x=1}^{z}\sum_{I\in C_{x}}{\left(I-P_{x}\right)}^{2}, \end{array}$$

where *i* is the element in cluster *C*_*x*_, *P*_*x*_ is the centre of cluster *C*_*x*_, and *z* is the number of clusters. In the process of K-means iteration, seek to minimize *Y*_*c*_. In the algorithmic idea of AC K-means, some dimensions of data can be used to describe all data structures. The dimension of data can be divided into two subspaces. One is m-dimensional subspace (clustering space), which contains all the structural information. The remaining d-m-dimensional space (noise space) does not contain any useful clustering structural information.

In order to obtain valuable spatial information and reduce the impact of useless information on clustering performance, the original data is mapped into two different subspaces and transformed as follows. Suppose there is an orthogonal matrix *Q*, which is used to map the original d-dimensional space to obtain the transformed *D* features. The first *m* features correspond to the clustering space, and the last (*d* − *w*) features correspond to the noise space. Therefore, projection will be carried out to achieve the purpose of space conversion.

(6) $$\begin{array}{c} U_{C}=\left[\begin{array}{c} X_{w}\\ 0_{d-w,w} \end{array}\right],\\ U_{T}=\left[\begin{array}{c} 0_{w,d-w}\\ X_{d-w} \end{array}\right], \end{array}$$

where *X*_*w*_ stands for the identity matrix with *w* × *w*. 0_*d*−*w*,*w*_ represents the zero matrix with (*d* − *w*) × *w*.

The way to map data I to cluster space is *U*_*C*_^*T*^*Q*^*T*^*I*. The way to map data I to noise space is *U*_*T*_^*T*^*Q*^*T*^*I*. Therefore, the sum of squares function of error in traditional K-means can be extended as follows:

(7) $$\begin{array}{c} Y_{c}=\sum_{x=1}^{z}\sum_{I\in C_{x}}{\left(U_{C}^{T}Q^{T}I-U_{C}^{T}Q^{T}P_{x}\right)}^{2}+\sum_{I\in S}{\left(U_{T}^{T}Q^{T}I-U_{T}^{T}Q^{T}P_{S}\right)}^{2}. \end{array}$$

*Y*_*c*_ consists of two parts. The former represents the information of clustering space, including the characteristics of the original space, and the other represents the information of noise space. What we need to do is to make the structure information of noise space as small as possible and the information of clustering space as large as possible, so as to achieve a balance between the two. By optimizing this objective function, we can find the optimal solution of K-means in the optimal subspace [15].

After the data is projected into the cluster space and noise space, the distance is no longer calculated by the Euclidean distance under the original dimension, but the projection *U*_*C*_^*T*^*Q*^*T*^*I* of the cluster space is used, that is, the nearest centre point is found in the subspace. The comparison formula is as follows:

(8) $$\begin{array}{c} Y={\text{arg}}_{x}\text{min}{\left(U_{C}^{T}Q^{T}I-U_{C}^{T}Q^{T}P_{x}\right)}^{2}. \end{array}$$

At the beginning of the algorithm, it is necessary to initialize the random orthogonal matrix *Q*, which can be obtained by singular value decomposition of any matrix, and *m* in *U*_*c*_ matrix can be set as *d*/2 for reference. In each iteration, keep the values of *Q*, w and *P*_*x*_ fixed, and assign each data point to the cluster with the smallest distance in the cluster space, to minimize the loss function in the form of cluster space.

### 2.3. Parameter Update

In K-means algorithm, only the centre point is updated after each iteration. In AC K-means, there are unknown parameters such as orthogonal matrix *Q*, clustering space dimension *m* and *S*_*x*_. So, it also needs to be updated during the execution of the algorithm. The symbols used below have the same meanings as those in Table 1.

For the centre point of the cluster, the update method in the traditional K-means is still used. The update method of orthogonal matrix *Q* will be given below.

First, fix the value of the dimension *w* of the clustering space, which is taken as *d*/2. In the K-means algorithm, the loss function is as follows:

(9) $$\begin{array}{c} Y_{c}=\sum_{x=1}^{z}\sum_{I\in C_{x}}{\left(U_{C}^{T}Q^{T}I-U_{C}^{T}Q^{T}P_{x}\right)}^{2}+\sum_{I\in S}{\left(U_{T}^{T}Q^{T}I-U_{T}^{T}Q^{T}P_{S}\right)}^{2}, \end{array}$$

*Y*_*c*_ can be minimized to a matrix eigenvalue decomposition problem.

(10) $$\begin{array}{c} Y_{c}=\sum_{x=1}^{z}\sum_{I\in C_{x}}{\left(U_{C}^{T}Q^{T}I-U_{C}^{T}Q^{T}P_{x}\right)}^{2}+\sum_{I\in S}{\left(U_{T}^{T}Q^{T}I-U_{T}^{T}Q^{T}P_{S}\right)}^{2}\\ =\sum_{x=1}^{z}\sum_{I\in C_{x}}{\left(U_{C}^{T}Q^{T}I-U_{C}^{T}Q^{T}P_{x}\right)}^{T}\left(U_{C}^{T}Q^{T}I-U_{C}^{T}Q^{T}P_{x}\right)\\ +\sum_{I\in S}{\left(U_{T}^{T}Q^{T}I-U_{T}^{T}Q^{T}P_{S}\right)}^{T}\left(U_{T}^{T}Q^{T}I-U_{T}^{T}Q^{T}P_{S}\right)\sum_{x=1}^{z}\sum_{I\in C_{x}}{\left(I-P_{x}\right)}^{T}QU_{C}U_{C}^{T}Q^{T}\left(I-P_{x}\right)+\sum_{I\in S}{\left(I-P_{S}\right)}^{T}QU_{T}U_{T}^{T}Q^{T}\left(I-P_{S}\right)\\ =\sum_{x=1}^{z}\sum_{I\in C_{x}}\text{Nr}\left({\left(I-P_{x}\right)}^{T}QU_{C}U_{C}^{T}Q^{T}\left(I-P_{x}\right)\right)+\sum_{I\in S}\text{Nr}\left({\left(I-P_{S}\right)}^{T}QU_{T}U_{T}^{T}Q^{T}\left(I-P_{S}\right)\right)\\ =Nr\left(U_{C}U_{C}^{T}Q^{T}\left[\sum_{x=1}^{z}\sum_{I\in C_{x}}\left(I-P_{x}\right){\left(I-P_{x}\right)}^{T}\right]Q\right)+\text{Nr}\left(U_{T}U_{T}^{T}Q^{T}\left[\sum_{I\in S}\left(I-P_{S}\right){\left(I-P_{S}\right)}^{T}\right]Q\right). \end{array}$$

Using the dispersion moment, it can be simplified as follows:

(11) $$\begin{array}{c} Y_{C}=\text{Nr}\left(U_{C}U_{C}^{T}Q^{T}\left[\sum_{x=1}^{z}S_{x}\right]Q\right)+\text{Nr}\left(U_{T}U_{T}^{T}Q^{T}S_{S}Q\right). \end{array}$$

It can be seen that *U*_*C*_*U*_*C*_^*T*^ is a diagonal matrix with the first *w* values of 1 and the last (*d* − *w*) elements of 0. *U*_*T*_*U*_*T*_^*T*^ is a diagonal matrix with the first *w* values of 0 and the last (*d* − *w*) elements of 1.

According to matrix knowledge, for any matrix *k*, if Nr(*U*_*C*_*U*_*C*_^*T*^*K*)=Nr(*K*) − Nr(*U*_*T*_*U*_*T*_^*T*^*K*), formula (12) can continue to be simplified as follows.

(12) $$\begin{array}{c} \text{Nr}\left(U_{C}U_{C}^{T}Q^{T}\left[\sum_{x=1}^{z}S_{x}\right]Q\right)+\text{Nr}\left(U_{T}U_{T}^{T}Q^{T}S_{S}Q\right)\\ =\text{Nr}\left(U_{C}U_{C}^{T}Q^{T}\left[\sum_{x=1}^{z}S_{x}\right]Q\right)-\text{Nr}\left(U_{C}U_{C}^{T}Q^{T}S_{S}Q\right)+\text{Nr}\left(Q^{T}S_{S}Q\right)\\ =\text{Nr}\left(U_{C}U_{C}^{T}Q^{T}\left(\left[\sum_{x=1}^{z}S_{x}\right]-S_{S}\right)Q\right)+\text{Nr}\left(Q^{T}S_{S}Q\right). \end{array}$$

For an orthogonal matrix *Q*, Nr(*Q*^*T*^*S*_*S*_*Q*) is a constant. Nr represents the trace of the matrix.

From the definition of *U*_*C*_, the upper left of *U*_*C*_*U*_*C*_^*T*^ is an *w* × *w* w identity matrix, and the values of the remaining elements are 0. And only *U*_*C*_ is related to *w*, the estimation of *Q* is not affected by *w* and the loss function is transformed to find the minimum of the matrix trace.

The eigenvectors of [∑_*x*=1_^*z*^*S*_*x*_] − *S*_*S*_ used here are used to update the transformation matrix *Q*, and the eigenvalues and eigenvectors of [∑_*x*=1_^*z*^*S*_*x*_] − *S*_*S*_ are solved first. The first *m* eigenvectors are inserted into the first *w* column of matrix *Q* and the last (*d* − *w*) eigenvectors are inserted into the last (*d* − *w*) column of matrix *Q* in order to obtain the new orthogonal transformation matrix *Q*.

In the generation process of subspace, the eigenvectors corresponding to the negative eigenvalues of [∑_*x*=1_^*z*^*S*_*x*_] − *S*_*S*_ are mapped to the cluster space, and the eigenvectors corresponding to the positive eigenvalues are mapped to the noise space. Therefore, the problem is equivalent to solving the minimization of the sum of all the negative eigenvalues. If there is no negative eigenvalue, the clustering subspace does not exist. W is 0, and the corresponding dataset S contains only one cluster. If the eigenvalue is zero, the effect on the loss function is uncertain. However, from the perspective of clustering, the clustering space tends to be smaller. Therefore, by projecting these eigenvectors into the noise space, the loss function of a given V can be optimized by setting *m* to the number of negative eigenvalues of [∑_*x*=1_^*z*^*S*_*x*_] − *S*_*S*_. Meanwhile, eigenvectors with negative eigenvalues close to zero (e.g., ≥1e-10) are expected to be assigned to noise space for the same reason as eigenvalues equal to zero.

## 3. System Design of This Paper

The software module of the design system mainly includes database module, functional Agent design module, and multi-agent collaboration module [16]. The specific design process is as follows.

### 3.1. Database Module

Database is not only the basis for the stable operation of the design system but also a part of the data storage of the design system. The database consists of data warehouse, model base, and knowledge base. Among them, data warehouse stores financial forecast plan, decision, control, and other related original information. The original information in the data warehouse is extracted from the accounting system, including cost, capital, sales, and profit. In order to facilitate the application of the design system, the original data information of the data warehouse is managed hierarchically. The details are shown in Figure 1.

As shown in Figure 1, the historical data layer is mainly time series data. Under normal circumstances, digital industry financial data of 5–10 years are stored. The current data layer stores the latest financial data of the digital industry. After a certain period of time, the design system will automatically transfer the data of this layer to the historical data layer. The summary data layer is to summarize the historical data and current data, and the obtained financial risk warning information is the comprehensive data needed for decision-making. The analysis and decision data layer refers to the highly comprehensive data, which can intuitively show the operating status of digital industries and help digital industry managers to make scientific and reasonable decisions.

Model base is one of the core parts of financial risk early warning information auxiliary decision system. It gathers all financial risk early warning models and stores all financial risk decision-making and analysis model description information [17]. The model library is mainly presented in the form of model dictionary. The details are shown in Table 2.

Knowledge base is a software system that supports knowledge generation, storage, maintenance, and invocation. It has functions such as search strategy, reasoning mechanism, access management, integrity, and consistency test.

### 3.2. Functional Agent Design Module

The functional Agent design module mainly consists of two parts, namely, interface Agent and information source Agent [4].

Interface Agent undertakes the task of human–computer interaction and runs through the whole decision-making process of financial risk warning information. The interface Agent structure is shown in Figure 2.

The information source Agent is the bridge between the financial risk early warning information auxiliary decision system and the network. Through the information source Agent, the design system can get financial information on the network, download, and store it, and enhance the accuracy of financial risk warning information. The Agent structure of information source is shown in Figure 3.

### 3.3. Multi-Agent Collaboration Module

The design system is composed of a group of independent and cooperative agents. Agent is the component unit of the design system and an independent entity. In the design system, the multi-agent realizes the financial risk warning task by cooperating with each other. Each Agent adjusts its own behaviour according to the information of itself and other agents to avoid conflicts.

The application of multi-agent cooperation mechanism is the widely used contract network model. The workflow is shown in Figure 4. In the contract network model, all agents are divided into two roles: manager and worker. In the multi-agent cooperation mechanism, the cooperation quality of multi-agent is mainly displayed through the parameters such as trust, friendliness, and positivity. Where trust refers to Agent *x*'s evaluation of Agent *y*'s ability to complete *u* tasks, denoted as Trust (*x*, *y*, *n*), and the initial value is set to 0.5.

When Agent *y* completes *n* type tasks, Agent *x*'s confidence in Agent *y* will increase Δ*C*_award_, and the expression is formula (13).

(13) $$\begin{array}{c} \text{ifevaluate}\left(x,y,n\right)>Q_{b}\text{ then Trust}\left(x,y,n\right)=\text{Trust}\left(x,y,n\right)+\Delta C_{\text{award}}. \end{array}$$

When Agent *y* fails to complete n-type tasks, agent *x*'s trust in it will be reduced Δ *C*_penalty_, the expression is formula (14).

(14) $$\begin{array}{c} \text{ifevaluate}\left(x,y,n\right)>Q_{l}\text{ then Trust}\left(x,y,n\right)=\text{Trust}\left(x,y,n\right)+\Delta C_{\text{penalty}}. \end{array}$$

Friendliness refers to the ratio of the number of tasks successfully completed by Agent *y* to the total number of tasks entrusted by agent *x*. The calculation formula is formula (15).

(15) $$\begin{array}{c} {\text{Friend}}_{\left(x,y,n\right)}=\frac{T_{\text{xy}}^{n}}{T_{y}^{n}}. \end{array}$$

Enthusiasm refers to the ratio of Agent *y* bidding times to all agent bidding times for the task sent by agent *x*. The calculation formula is formula (16).

(16) $$\begin{array}{c} \text{Active}\left(x,y,n\right)=\frac{T_{y}^{n}}{\sum_{z=1}^{t}T_{z}^{n}}. \end{array}$$

According to the bidding and task completion of each Agent, the design system manager can modify its parameters in real time to ensure the efficient completion of the design system. Through the design of hardware unit and software module above, this paper realizes the operation of financial risk early warning information auxiliary decision system, which provides certain help for the development of Chinese digital industry and financial risk early warning research.

## 4. Experiment and Analysis

The dataset used in the experiment contains 10 years of real trading data, which includes more than 30 million trades made by 25,000 traders. The missing values were replaced using EM interpolation and the outlier processing of literature [18]. Supervised learning requires a labelled dataset *D*={*j*_*x*_, *i*_*x*_}_*x*=1,…,*t*_, where *i*_*x*_ is the feature vector representing transaction *x*, *j*_*x*,_ is the target variable. Use information from previous trades to decide whether to hedge the current trade. If the target variable *j*_*x*,_ is set to 1, it indicates that a hedging strategy is adopted, and if it is set to -1, it indicates that no hedging strategy is adopted. When  return_*x*_ is greater than or equal to 5%, *j*_*x*,_ is equal to 1. Otherwise, *j*_*x*_ is equal to minus 1. The calculation method of returni is as follows.

(17) $$\begin{array}{c} {\text{return}}_{x}=\frac{\sum_{20<y⩽100}{\text{UL}}_{\text{xy}}}{\sum_{20<y⩽100}M_{\text{xy}}}\circ \circ \circ , \end{array}$$

where UL_xy_ is the profit and loss of transaction *y*, and *M*_xy_ is the amount required by the market maker to place the order. Compare this algorithm with Literature [19], Literature [20], and Literature [21].  Table 3 shows the comparison of the four classification algorithms under multiple evaluation criteria. The results in Table 3 are obtained by averaging the results of 10-fold cross-validation. According to the performance indicators in Table 3, the algorithm in this paper is superior to other algorithms.

To clarify the value of deep structure, the proposed algorithm is compared with Literature [22], which removes the network of deep hidden layers.  Figure 5 shows the ROC curve and Figure 6 shows P-R(Precision-Recall) curve of the algorithm and Literature [22] in this paper. According to the ROC Curve, the AUC of the algorithm in this paper is larger, which means that the algorithm in this paper has high accuracy. Combined with the results of the P-R curve, the deep architecture can improve the classification ability of the network.

Next, the performance of unsupervised pretraining stage is investigated. The purpose is to judge whether the algorithm in this paper can learn the distributed representation that can distinguish a-book and b-book customers in unlabeled data.  Figure 7 shows the curve of activation value. Results show that when a transaction is received from a b-book customer, the activation value is often less than 0.4, and the transaction of a-book customer usually causes the activation value to be greater than or equal to 0.4.

In order to further verify the performance of this algorithm in financial risk early warning of large-scale digital industries, 1318 alarm data of 100 listed digital industries are analyzed by using literature [23], literature [24], literature [25], and proposed algorithm. The simulation results are shown in Figure 8.

From Figure 8, we can see that the early warning accuracy of the algorithm in this paper is the highest, followed by literature [25], and literature [23] is the worst. In terms of early warning time performance, the algorithm of literature [23] is the best, the algorithm of literature [24] and the algorithm in this paper are the second, and the algorithm of literature [25] is the worst. Comprehensive comparison shows that this algorithm has better performance in dealing with large-scale digital industry sample early warning.

## 5. Conclusion

The financial crisis continues to break out all over the world, and its frequency and destructiveness are increasing. In the face of massive unstructured data, the field of digital industry financial risk warning is faced with many challenges. It is of great significance to extract valuable information accurately and effectively for risk warning from mixed multisource, heterogeneous, and high-frequency data. In order to discover digital industry financial risks in time and give early warning, this paper proposes an early warning system of corporate financial risks based on improved K-means clustering algorithm. In order to speed up the K-means calculation and find the optimal clustering subspace, a specific transformation matrix is used to project the data. The feature space is divided into clustering space and noise space, the former contains all spatial structure information, the latter does not contain any information. Using the idea of spatial projection, the feature is divided into clustering space and noise space by transformation matrix. Compared with the original space, the clustering space information density of the proposed algorithm is higher and the dimension is smaller. It can reduce the time consumption of each distance calculation by K-means and achieve the effect of reduction and feature screening. The algorithm proposed in this paper has relatively broad application scenarios, and can work well in the case of obscure clustering spatial structure, and does not require prior information such as categories. However, when the dimension of data features is high and sparse, the algorithm in this paper may not be able to find the optimal subspace, which is also the direction of further optimization.

## Figures and Tables

**Figure 1:** Original data information hierarchy management framework.

**Figure 2:** Structure diagram of interface Agent.

**Figure 3:** Structure diagram of information source Agent.

**Figure 4:** Work flow chart of contract network model.

**Figure 5:** The curve of ROC.

**Figure 6:** The curve of P-R.

**Figure 7:** The curve of activation value.

**Figure 8:** Performance curve of digital industry financial risk early warning with different algorithms.

**Table 1:** Symbol conventions.

Symbol	Explain
*d* ∈ *T*	Number of dimensions of original data
*w* ∈ *T*	Number of dimensions of cluster space
*z* ∈ *T*	Number of clusters
S	A collection of all data
*Cx*	A collection of data in cluster x
*I* ∈ R	D-dimensional data
*P*_*S*_ ∈ **R**^*d*^	Centre of dataset s
*P*_*x*_ ∈ **R**^*d*^	Centre of cluster x
*S*_*S*_ ∈ **R**^*d*×*d*^	Scatter matrix of dataset *s* in original space
*S*_*x*_ ∈ **R**^*d*×*d*^	Scatter matrix of family *X* in primitive space
*P*_*C*_ ∈ **R**^*w*×*d*^	Mapping matrix of clustering space
**U**_*t*_ ∈ **R**^*d*−*w*×*d*^	Mapping matrix of noise space
Q	Random orthogonal matrix
*X*_*l*_	Identity matrix of LXL dimension
O_*x*,*r*_	Zero matrix of LXR dimension

**Table 2:** Model dictionary.

Data item	Explain	Remarks
Model number	Natural sequence number	Model dictionary primary key
Model name	Data model name	—
Body number	Model decision subject	Non-primary key
Model function	Detailed description	Object, condition, and function
Mathematical description	Mathematical formula	Mode storage with formula editing function
Constraint condition	Application conditions	—
Design language	Programming form	For example, VB
Executable program	Solver code	Binary file storage
Input/output parameters	Input parameter list	Define the man–machine interface output mode and storage mode
Parent/child model	List	Not fixed/relatively fixed
Model log	Model call topics and times	—

**Table 3:** Performance comparison of classification algorithms.

Algorithm type	Profit and loss/yuan	Misclassification cost/yuan	Sensitivity index	Accuracy
Proposed	1120.47	4386.59	0.652	0.994
Literature [19]	1007.47	8281.46	0.321	0.985
Literature [20]	936.24	8477.61	0.305	0.974
Literature [21]	639.54	7468.29	0.392	0.976

## Data Availability

The labelled datasets used to support the findings of this study are available from the corresponding author upon request.
